The article "Analysis of the Effect of Nursing Intervention on Children with Respiratory Tract Infection Based on Comprehensive Nursing" was retracted in 2022. Reason: concerns about the peer review.

# Analysis of the Effect of Nursing Intervention on Children with Respiratory Tract Infection Based on Comprehensive Nursing

**DOI:** 10.1155/2021/6923823

**Published:** 2021-09-15

**Authors:** Yujie Chen, Qing Li

**Affiliations:** Shengjing Hospital of China Medical University, Shenyang, Liaoning, China

## Abstract

Recurrent respiratory tract infections in children are common. It means that children are repeatedly exposed to external pathogens within a certain time, and the clinical symptoms are reciprocating. This article carries out nursing intervention on children's respiratory tract infection through comprehensive nursing methods and analyzes the intervention effect. Moreover, this paper uses a controlled trial to study the nursing methods of recurrent respiratory tract infections in children. In addition, this paper determines and screens test samples according to relevant standards, conducts different nursing methods on samples of different groups, and compares them with the same indicators. Finally, this paper combines mathematical statistics to make statistics of experimental results and draws tables and statistical graphs. By comparing multiple parameters, it can be seen that the comprehensive nursing intervention has a good effect on the nursing of children with respiratory tract infection compared with the traditional nursing intervention, so this nursing method can be expanded in the future.

## 1. Introduction

The exact pathogenesis of RRTI in children is still unclear. At present, it is considered that the comprehensive action of multiple factors causes the disease. In addition to infection factors, it is also related to immunodeficiency or hypofunction, respiratory tract anatomy, congenital and chronic diseases, nutritional disorders, improper treatment, heredity, and upbringing. Among them, immunodeficiency is an important reason for RRTI. To prevent children from suffering from RRTI, improving immunity is the focus of prevention and treatment. However, the development of the immune system of infants and young children is not yet mature, and the immune globulin provided by the mother decreases after six months, so the chances of disease are relatively increased. In addition, multiple pathogen infections can lead to immune fatigue in children, which leads to further deterioration of immune function in children and makes children more susceptible to infection. RRTI is often the case that old diseases have not healed and new feelings have reappeared and repeated over the years, which can easily lead to nutritional disorders. As a result, a vicious circle of “nutrition disorders-low immune function-repeated infections-aggravated nutritional disorders” is formed.

The article "Analysis of the Effect of Nursing Intervention on Children with Respiratory Tract Infection Based on Comprehensive Nursing" was retracted in 2022. Reason: concerns about the peer review.

The growth and development of children is the result of the interaction between genetics and environmental factors, including nutrition, disease, economy, and culture. Infants and young children are less affected by genetics and are more susceptible to nutrition, disease, feeding methods, and medical nursing. During the whole process of recurrent respiratory tract infections and difficult recovery in children with RRTI, the body's energy consumption is higher than that of healthy children, and the disease itself and repeated use of drugs may cause loss of appetite, poor digestion, and absorption, resulting in insufficient nutrients. In addition, the reduction of outdoor activities in children with RRTI affects the synthesis of vitamin D, and the disease also affects the quality of sleep to a certain extent. Therefore, it is urgent to carry out further research to explore scientific and reasonable targeted intervention measures.

Most research on children's RRTI focuses on the etiology, diagnosis, therapy, and other aspects of the condition. Still, there are few studies on the effect of children's RRTI on physical development and children's RRTI intervention. Internal variables such as allergies, atopy, preterm delivery, and low birth weight and external ones such as feeding practices, malnutrition, vaccination, and living environment may all contribute to a child's RRTI. It helps prevent RRTI or decrease the incidence of RRTI, relieve the illness, and shorten the course of the disease by avoiding or modifying certain changeable risk factors. Traditional Chinese medicine's views on illness prevention are comparable to Western medicine's preventive ideas. Traditional Chinese medicine treats children differently depending on their physical characteristics. As a result, Chinese medicine has general conditioning features that vary from person to person. Chinese and Western medicine have distinct features in terms of illness prevention. Different approaches may be utilized to enhance the effectiveness of interventions based on the unique circumstances of children. We address the symptoms of the illness when it is more urgent, and the root of the disease when it is less urgent, so that RRTI may be better avoided.

Based on the above analysis, this paper carries out nursing intervention on children's respiratory tract infection through comprehensive nursing methods and analyzes the effect of intervention.

## 2. Related Work

Literature [1] has done some investigations on the growth and development of children with recurrent respiratory tract infections. Literature [2] implemented physique intervention on children through community intervention, which reduced the incidence of children's RRTI and alleviated the condition. Literature [3] mentioned the risk factors of children's RRTI in the “Practical Guidelines for the Diagnosis and Management of Children's RRTI.” It emphasized the importance of prevention in managing children's RRTI. Literature [4] found in a survey that French general practitioners support adopting a preventive approach to manage RRTI in children.

The article "Analysis of the Effect of Nursing Intervention on Children with Respiratory Tract Infection Based on Comprehensive Nursing" was retracted in 2022. Reason: concerns about the peer review.

Literature [5] found that the incidence of RRTI in children with congenital cleft lip and palate and foreign bodies in the bronchus was significantly higher than that of normal children. Thus, it can be seen that although the incidence of congenital anatomical abnormalities in children with RRTI is low, it is not uncommon. According to the physiological and anatomical characteristics of the respiratory tract in children, it is found that the child's respiratory tract is narrow. In addition, there is a low air volume, insufficient lung elastic fibers, incomplete development of the body's respiratory system, and imperfect functions.

Moreover, children's mucosal lymphatic vessels are richer, and the tissues are delicate and soft, so they are more sensitive to external stimuli and lack disease resistance. Therefore, the specific and nonspecific functions of the respiratory tract are poor. Once the infection occurs, it is easy to cause local mucosal edema and cause respiratory symptoms. In addition, RRTI caused by respiratory obstruction caused by acquired factors cannot be ignored and needs clinical attention. There are clinical reports that the high incidence of bronchial foreign bodies in children is 1–3 years old, mainly related to the children's youngness, lack of self-control and self-protection ability, and crying, laughing, and playing when eating. In addition, the teeth are underdeveloped, some hard foods cannot be chewed carefully, and the chewing and swallowing functions of infants and young children are not coordinated. Furthermore, the cough reflex is not fully developed [6].

Literature [7] found that children's irregular use of broad-spectrum antimicrobial drugs makes bacteria continue to increase drug resistance under selective pressure. Studies have shown that the drug resistance of common pathogenic bacteria in the respiratory tract of children is increasing year by year. This is related to the excessive use of antibiotics because of some hospitals and parents' eagerness for success and blind pursuit of pure curative effect. In addition, due to the weak national food hygiene supervision, some food manufacturers add many antibacterial drugs in the breeding process to reduce the prevalence of animal husbandry. These have greatly promoted the production of drug-resistant bacteria, reduced the efficacy of antibacterial drugs, and caused unhealed respiratory infections in children [8].

The article "Analysis of the Effect of Nursing Intervention on Children with Respiratory Tract Infection Based on Comprehensive Nursing" was retracted in 2022. Reason: concerns about the peer review.

From the perspective of the law of life development, children have the fastest growth and development speed as the early stages of life. Compared with adults, children need more nutrients in their bodies [9]. However, its imperfect digestive organs and functions make it difficult to meet the body's needs for trace elements, vitamins, and other substances. These substances are just the “nutrients” needed by the human body to exert immune function. If the body lacks these important substances, it can lead to weakened immune function [10]. When the concentration of a certain trace element in the body is low, malnutrition can lead to growth retardation or obstacles and a decline in immune function. Literature [11] shows that the levels of trace elements in children with RRTI are significantly lower than those in healthy children, related to the frequency of attacks and the severity of the disease. In modern society, most single children are valued by the whole family. To meet their children's requirements, parents will inevitably overindulge their children. The recurrence of part of the relapsed infants is due to partial eclipse, picky eaters, eating too many snacks and frozen foods, and not forming a good eating habit and balanced diet structure, resulting in a lack of trace elements in the body, impaired gastrointestinal function, and low immunity [12].

Because children with RRTI will have repeated episodes of disease, they need to see a doctor frequently, which affects the children's normal study and life, and will have a greater impact on their psychology [13]. Literature [14] shows that the detection rate of abnormal psychological behavior of children with RRTI is significantly higher than that of the control group through psychological research on children with RRTI. Frequent mental stress can cause frequent RRTIs. Literature [15] found through investigation that the psychological stress score of children with RRTI was higher than that of the control group, and children with high psychological stress were more likely to suffer from repeated respiratory infections.

Literature [16] shows that the condition of the children in the RRTI group is significantly reduced after supplementation of trace elements. Literature [17] regarded children with RRTI as the observation group and normal healthy children as the control group. The study found that the trace elements such as calcium, zinc, copper, and humoral immune factors in children with RRTI were lower than those in the control group. These trace elements are the important substances involved in synthesizing various nucleic acids and proteins of the human body and repairing cell tissues. In addition, humoral immune factors such as IgG have important functions such as activating immune cells, killing pathogenic microorganisms, neutralizing endotoxins, and regulating the function of phagocytes. Literature [18] used zinc gluconate tablets to follow-up children with recurrent upper respiratory tract infections. They found that oral zinc gluconate tablets can supplement trace elements, enhance the children's resistance, and reduce recurrence.

The article "Analysis of the Effect of Nursing Intervention on Children with Respiratory Tract Infection Based on Comprehensive Nursing" was retracted in 2022. Reason: concerns about the peer review.

Literature [19] found that, after using mental relaxation therapy, children with RRTI's condition were reduced, and at the same time, the psychological and emotional conditions are improved to a certain extent. In addition, in the treatment process, children often cannot understand the language of medical staff due to psychological fear, resulting in low compliance with treatment and delay in diagnosis and treatment. Literature [20] advocated that strengthening psychological comfort through physical movements can effectively improve children's compliance with respiratory infections, thereby enhancing the treatment effect and preventing complications.

Literature [21] shows that IgG and its subtypes in children with RRTI are significantly lower than those in healthy children. After treatment, the level of IgG increases, which reduces the incidence of RRTI, reduces symptoms, and shortens the course of the disease. Children with RRTI have defects in immune function and abnormal pulmonary ventilation, so the respiratory tract is susceptible to infection by pathogenic microorganisms, and the airway mucosa is prone to inflammation and hyperresponsiveness, causing a vicious circle.

## 3. Objects and Methods

The cases were all from children admitted to a hospital from December 2018 to December 2020, with a total of 100 cases. The informed consent process complies with the regulations, the legal guardians signed the informed consent form, and the children meet the inclusion criteria.

Western medicine diagnostic criteria: the criteria are according to the “Clinical Concepts and Management Principles of Recurrent Respiratory Tract Infections” revised by the Respiratory Group of the Pediatric Branch of the Chinese Medical Association and the Editorial Committee of the Chinese Journal of Pediatrics (Table 1) [22].

Case selection criteria: case inclusion criteria meet the diagnostic criteria for recurrent respiratory infections. The selection age is 1 to 3 years. Moreover, the acute infection recovered within 1 week. Therefore, the course of the disease is at least 1 year. In addition, the informed consent process complies with regulations, and the legal guardian signs the informed consent form [23].

The article "Analysis of the Effect of Nursing Intervention on Children with Respiratory Tract Infection Based on Comprehensive Nursing" was retracted in 2022. Reason: concerns about the peer review.

Exclusion criteria: children with severe primary respiratory tract infections such as primary or acquired immunodeficiency syndrome, respiratory malformations, congenital heart disease, and gastroesophageal reflux disease are excluded. Children who used immunomodulators and other drugs to treat recurrent respiratory infections in the past year are excluded. Children with severe primary disease in each system are excluded. Children with allergies or allergies to the ingredients of the preparation are excluded. Children who could not cooperate or were participating in other drug trials were excluded. According to the investigator's judgment, children who are likely to be lost to follow-up are excluded.

Remove criteria: children who had allergic reactions, serious adverse events, and complications and the investigators judged that the trial should be stopped are removed from the test. Children with other diseases that affected the efficacy and safety are removed from the test during the trial. Children with poor compliance, automatic dressing change, or addition of Chinese and Western medicines prohibited by this plan are removed from the test. During the test, children with respiratory tract infection and the drug is stopped for more than 10 days are removed from the test. For whatever reason, the child or the child's parent is unwilling or impossible to continue the clinical trial being removed [24].

Rejection criteria: children who seriously violated the inclusion or exclusion criteria are rejected. Children who had not taken medication after enrollment are rejected. Children who are automatically lost to follow-up and had no posttreatment visit records are rejected.

We observe and analyze the role of comprehensive nursing methods in recurrent respiratory tract infections in children and compare them with the control group of traditional nursing methods to objectively evaluate its clinical efficacy. At the same time, we apply comprehensive nursing to treat children with RRTI to help reduce the incidence of respiratory infections.

The 100 children with RRTI who met the inclusion criteria are divided into a test group and a control group according to the parents' wishes, and each group includes 50 samples [25].

The control group received routine emergency nursing. First, the nursing staff adjusts the child to a prone position. It should be noted that the child should not be moved at will. Afterward, the nursing staff unifies their clothes and turns their heads to one side to immediately remove foreign bodies in the respiratory tract and keep the respiratory tract unobstructed. If the convulsions are severe, the nursing staff can place gauze in their oral cavity. A fence should be installed around the bed to prevent falling out of the bed. After the children's physical signs are stable, the nursing staff will give oral education to the family members, keep the room temperature and humidity appropriate, and reduce the number of visits. The observation group is given comprehensive nursing. (1) Cool down: ① first, the nursing staff adjust the indoor temperature to 20°C–22°C and the humidity to 50%–60% and open the windows for 30 minutes to ventilate. After that, the nursing staff places the ice pack on the neck, armpits, forehead, and headrest ice pack and replaces them regularly or wipes the child's body with 30%–40% ethanol or 32°C–36°C warm water. If the physical cooling effect is not good, the hibernation mixture can be used together. Drug intervention, first, the nursing staff establish intravenous access and give diazepam according to the doctor's order. The dose is 0.3–0.5 mg/kg each time, and the enema is retained. The buttocks are raised during the enema so that the child can fully absorb the drug. ② After 0.5 h of intervention, the nursing staff need to measure the patient's body temperature regularly. If the rectal temperature drops to 38.5°C and the axillary temperature drops to 38°C, it indicates that the cooling effect is effective. If the body temperature rises with symptoms such as mental changes, lymphadenopathy, and abdominal pain, nurses need to inform the doctor immediately. (2) Skin: the nursing staff need to wipe the children's body with warm water on time, keep the skin clean and dry, change clothes and sheets in time, and observe the degree of sweating. If the child loses too much sweat, fluids can be supplemented. (3) Oral cavity: the nursing staff assists the children to rinse their mouths with normal saline or uses sodium chloride solution (with a concentration of 0.9%) to wipe their mouths. There is a need to apply paraffin oil to the children regularly to prevent dryness of the mouth and at the same time do a good job of oral cleaning. (4) Convulsions: once the child has a seizure, the nursing staff removes the pillow and tilt the child's head in one direction. It is important to note that children cannot be moved arbitrarily. At the same time, the nursing staff helps the patient clean up the secretions in the oral cavity to not affect breathing. The nursing staff can use tongue forceps to slightly pull the tongue out for children with recurrent seizures to avoid falling behind the tongue. (5) Oxygen nursing: the nursing method is adjusted according to the age of the child. The younger child is given oxygen inhalation with a mask, and the oxygen flow per minute is controlled at 4-5 L. For older children, oxygen inhalation with nasal cannula is used, and the oxygen flow rate is controlled at 1-2 L per minute. (6) Basic nursing: the nursing staff will provide health education to the children's family members, relieve their worries, and inform them that the children should refrain from drinking in time when the children have convulsions, and they can resume eating after the condition is controlled. Moreover, children should rinse their mouths with warm water after eating and frequently wash and change their clothing. In addition, the nursing staff need to instruct children to do simple housework to strengthen physical exercise and improve resistance.

The article "Analysis of the Effect of Nursing Intervention on Children with Respiratory Tract Infection Based on Comprehensive Nursing" was retracted in 2022. Reason: concerns about the peer review.

The children in the observation group received comprehensive nursing interventions on the routine nursing model. First, the ward environment is effectively controlled, and the room temperature is adjusted according to the actual degree of the child's illness. The temperature is controlled at about 18–22 degrees Celsius, and the humidity is controlled at 55%. At the same time, nurses should also conduct regular ventilation and disinfection treatments to ensure the effectiveness of indoor air circulation. The children's favorite cartoons are played in the ward to divert their attention and stabilize their treatment emotions. Secondly, the patient's condition is tested, and the child's body temperature is measured every four hours. If sudden changes are found, the nursing staff will immediately record and take effective intervention measures to intervene.

Moreover, nurses need to conduct a comprehensive assessment of the patient's condition, communicate with the doctor in time if other special problems are found, and take targeted treatment measures. In addition, it is often difficult for children to get a good rest when their body temperature is too high. Therefore, the nursing staff should pay attention to monitoring changes in the child's body temperature. When the child sweats, it should be wiped off immediately, and the clothes should be changed in time. When the body temperature is higher than 38 degrees, medication and physical forms should be taken immediately to cool down. Based on the psychological level, nurses also need to carry out all-round intervention. That is, the nursing staff should communicate with the patient's family members and effectively assist the nursing staff in venting the negative emotions of the patient. There is a need to improve the family's confidence in treatment based on related successful treatment cases and encourage them to encourage the child to cooperate with the treatment. In addition, the nursing staff need to make relevant nursing interventions for infection prevention and health guidance. For example, when upper respiratory tract infections are common, the children's nutrition and physical exercise should be appropriately improved. The hospital environment and the patient's clothing should be adapted according to the climate and other differences.

The article "Analysis of the Effect of Nursing Intervention on Children with Respiratory Tract Infection Based on Comprehensive Nursing" was retracted in 2022. Reason: concerns about the peer review.

For all children, emergency treatment is given, and the emergency treatment methods include acupuncture and acupoint pressing. Moreover, the nursing staff needs to perform stimulating activities by pressing on the pediatric hyperfebrile convulsion patient. Subsequently, the nursing staff needs to use the intravenous injection of phenobarbital sodium to provide analgesic treatment to patients with pediatric convulsions and quickly improve tissue hypoxia while ensuring that the airway remains unobstructed. After that, the nursing staff administered an intramuscular injection of dexamethasone to cool the children and gave mannitol to dehydration of the children with convulsions. Comprehensive emergency nursing is carried out after preparations are made, and the specific methods are as follows. First, the nursing staff provides high fever nursing for children with febrile seizures. By following the doctor's advice, the nursing staff takes medication to lower the temperature. If the patient's body temperature exceeds 39 degrees, the nursing staff can take physical cooling and use ice packs and wet towels to ice the armpits, groin, and other parts to reduce the fever. During the process, the nursing staff can also observe the relevant changes in body temperature. If the body temperature of children with convulsions and high fever drops to normal body temperature, the ice pack can be stopped. For the warm water bath, the general temperature is between 32 degrees and 36 degrees. By rubbing the skin more, the body temperature of children with febrile seizures can be reduced. The application of antipyretics is oral, and intramuscular injection of dexamethasone can also be used. Second, the treatment of convulsions is as follows. When a child has a seizure, the nursing staff should tilt the child's head to the other side to effectively deal with the secretions of the oral and nasal cavity. Moreover, nurses need to place related items between the upper and lower molars of the child, such as a tongue depressor, to avoid biting themselves due to a convulsive seizure. After the breathing of children with febrile seizures is restored, the flow of oxygen should be adjusted.

At the same time, the changes in consciousness and pupils should be observed during the process. If there is no obvious change in the child's pupil, it is used as the evaluation standard for transient convulsions. When the pupil size changes for a long time, the doctor should be notified immediately for rescue. The third is to reduce stimulation. Due to the strong light and loud noise in the ward, such phenomena should be effectively avoided during treatment. At the same time, concentrated operations should be carried out to avoid unnecessary stimulation. The fourth is to closely monitor the vital signs of children. The physical signs of children with high fever have various changes, and their pupils and consciousness are a reaction to their own condition. Therefore, the vital signs should be recorded in detail, and the type and interval of convulsions in children with febrile seizures and related conditions should be recorded. If an abnormality is found, it should be dealt with in time.

The article "Analysis of the Effect of Nursing Intervention on Children with Respiratory Tract Infection Based on Comprehensive Nursing" was retracted in 2022. Reason: concerns about the peer review.

## 4. Results

Through the above-controlled experiments, this paper researches the role of comprehensive nursing intervention in the nursing of children with respiratory tract infections. The comparison of treatment-related indicators between the two groups of patients is statistically compared. The cooling and hospitalization times are shown in Table 2, Figure 1, Table 3, and Figure 2, respectively.

In the comprehensive nursing of this paper, when a convulsion occurs, the nursing staff remove the pillow and tilt the child's head in one direction. At this time, the nursing staff should not move the child arbitrarily and need to help the patient clean up the secretions in the oral cavity to not affect the breathing. For children with recurrent seizures, nurses can use tongue forceps to slightly pull the tongue out to avoid falling behind the tongue. After that, this paper counts the convulsion control time and user satisfaction, and the results are shown in Table 4, Figure 3, Table 5, and Figure 4.

## 5. Analysis and Discussion

This study found that the text group's symptoms disappeared, the hospital stay is shorter than the control group, the nursing satisfaction is higher than that of the control group, and the recurrence rate is lower than that of the control group. It is suggested that comprehensive nursing can speed up the recovery process of children with febrile convulsions caused by upper respiratory tract infection, improve nursing satisfaction, and reduce the recurrence of convulsions. The reason is that comprehensive nursing takes the degree of nursing as the core of nursing work, which is a systematic nursing method. Moreover, it emphasizes the integrity of nursing, integrates the advantages of clinical nursing, and enhances the nursing effect. In addition, it improves the symptoms by strengthening the temperature control of the children. Therefore, comprehensive nursing is an important part of treating children with febrile seizures caused by upper respiratory tract infection. Based on conventional first aid measures, these nursing measures are further refined to improve clinical symptoms, speed up the recovery process, and enhance nursing satisfaction. Compared with conventional nursing, it is more targeted and comprehensive. Moreover, comprehensive nursing provides routine check-ups for children and includes a number of systemic nursing methods so that they can receive more comprehensive nursing services. The condition of febrile convulsion caused by upper respiratory tract infection in children is critical, so careful nursing and timely emergency measures to cool down are important prerequisites for treating children. This nursing takes cooling measures as a key measure. It cooperates with oral and skin nursing based on cooling measures to effectively control symptoms such as convulsions and high body temperature to minimize damage to the human body. An ice pack placed on the head can improve the hypoxia tolerance of brain tissue, reduce brain tissue metabolism, and relieve cerebral congestion. At the same time, timely replacement of ice packs can effectively avoid head frostbite. Ethanol wiping takes advantage of the volatilization of alcohol to speed up the heat dissipation of the skin, expand blood vessels, and increase heat dissipation, especially suitable for young children. In addition, comprehensive nursing requires nursing staff to do daily preventive work, cultivate good hygiene habits for children, strengthen nutritional intake and physical exercise, enhance the body's resistance to viruses and bacteria, and prevent recurrence from the source of the disease. In addition, the use of comprehensive nursing promotes nursing staff to have good observation and initiative. By strengthening the observation of the condition, the signs of recurrence of symptoms can be discovered in time, so that symptomatic measures such as oxygen inhalation can be implemented in a predictive manner. Moreover, potential safety hazards can be eliminated in time to control the condition as soon as possible, maintain the physical and mental comfort of the child, speed up the improvement of symptoms, shorten the length of hospitalization, and help improve nursing satisfaction.

The article "Analysis of the Effect of Nursing Intervention on Children with Respiratory Tract Infection Based on Comprehensive Nursing" was retracted in 2022. Reason: concerns about the peer review.

Finally, timely and effective intervention treatment and nursing of the disease are particularly important. At present, the actual compliance effect of most children in receiving treatment and nursing is not ideal, and some children even have psychological resistance. The intervention model based on comprehensive nursing is a series of nursing measures around children. It fully considers children's psychological development characteristics, such as immaturity, and creates a good treatment atmosphere for them. Psychological education and health promotion effectively reduce complications and disease recurrence in children and improve clinical treatment effects. This study showed that the length of hospitalization and antipyretic time of the patients in the actual observation group were reduced compared with the control group, and the complications of the patients were significantly reduced. Thus, it can be seen that comprehensive nursing intervention has a good effect on children with repeated respiratory infections. In addition, based on the satisfaction of patients and their relatives with the nursing and the general support of the observation group of patients for the nursing model, it can be explained that the nursing model has high applicability and promotion value.

## Figures and Tables

**Figure 1:** Statistical diagram of the cooling time of the test group and the control group.

**Figure 2:** Statistical diagram of hospitalization time of the test group and the control group.

**Figure 3:** Statistical diagram of convulsion control time (d) of the test group and the control group.

**Figure 4:** Statistical diagram of nursing satisfaction of the test group and the control group.

**Table 1:** Judgment conditions of recurrent respiratory tract infections in children.

Age	Recurrent upper respiratory tract infection (times/year)	Recurrent lower respiratory tract infections (times/year)	
		Recurrent tracheal and bronchial inflammation	Recurrent pneumonia
0–2	7	3	2
2–5	6	2	2
Over 7 years old	5	2	2

**Table 2:** Statistical table of cooling time of test group and control group.

No.	Control group (H)	Test group (H)	No.	Control group (H)	Test group (H)
1	70.7	41.6	26	70.2	42.5
2	75.2	50.0	27	80.0	44.1
3	73.3	42.1	28	77.7	41.7
4	77.5	48.7	29	76.1	49.1
5	77.8	45.9	30	74.5	44.7
6	78.6	47.0	31	71.3	42.6
7	79.9	45.1	32	73.2	49.1
8	75.5	47.3	33	78.9	49.2
9	77.6	44.6	34	71.7	45.4
10	75.0	41.8	35	79.6	46.1
11	73.8	45.5	36	79.4	41.3
12	78.0	42.1	37	74.0	45.7
13	75.3	41.2	38	73.2	48.3
14	70.5	44.0	39	76.9	42.3
15	76.5	42.5	40	76.6	48.4
16	75.5	40.8	41	76.2	43.8
17	71.7	47.9	42	75.7	44.7
18	70.5	48.9	43	72.1	46.0
19	78.1	46.9	44	74.0	44.6
20	71.1	42.5	45	75.6	40.4
21	74.3	46.1	46	78.2	42.7
22	70.2	40.5	47	79.0	46.1
23	71.0	43.5	48	75.5	42.7
24	79.4	49.1	49	74.8	43.2
25	72.5	44.1	50	75.2	49.2

**Table 3:** Statistical table of hospitalization time of the test group and the control group.

No.	Control group (H)	Test group (H)	No.	Control group (H)	Test group (H)
1	21.5	13.5	26	20.4	14.5
2	20.0	12.2	27	19.4	14.0
3	20.8	12.9	28	22.7	13.5
4	20.1	13.1	29	22.9	12.2
5	22.8	14.1	30	19.2	13.0
6	19.5	12.8	31	22.7	14.5
7	22.1	13.5	32	21.5	12.0
8	22.7	12.8	33	22.4	12.8
9	21.4	14.6	34	22.8	12.3
10	20.8	14.8	35	19.7	13.0
11	19.9	14.0	36	20.7	13.0
12	21.4	13.8	37	19.0	12.6
13	22.7	13.7	38	20.1	14.0
14	19.2	13.3	39	21.5	12.6
15	19.4	13.9	40	20.5	13.6
16	21.4	13.5	41	21.3	12.5
17	20.5	15.0	42	21.3	13.3
18	20.8	13.6	43	20.2	13.4
19	22.3	14.8	44	22.3	13.3
20	21.8	12.6	45	22.6	12.8
21	22.3	13.1	46	21.8	12.8
22	22.5	13.4	47	20.3	13.4
23	22.5	12.8	48	21.8	12.2
24	22.6	13.4	49	20.8	13.3
25	22.1	12.3	50	22.7	14.4

The article "Analysis of the Effect of Nursing Intervention on Children with Respiratory Tract Infection Based on Comprehensive Nursing" was retracted in 2022. Reason: concerns about the peer review.

**Table 4:** Statistical table of convulsion control time (d) of the test group and the control group.

No.	Control group (D)	Test group (D)	No.	Control group (D)	Test group (D)
1	6.18	3.78	26	6.17	3.84
2	5.24	3.70	27	5.22	4.08
3	5.12	4.42	28	5.39	4.20
4	5.27	4.38	29	5.37	3.74
5	5.07	4.27	30	5.86	3.96
6	6.18	3.51	31	5.15	3.68
7	5.78	4.02	32	5.15	4.34
8	5.69	3.51	33	6.16	4.34
9	5.62	3.85	34	5.49	4.41
10	5.89	3.72	35	5.11	3.77
11	6.25	4.23	36	6.24	4.46
12	6.14	4.30	37	6.33	3.81
13	5.42	3.55	38	6.23	4.36
14	6.47	4.44	39	5.12	3.90
15	6.30	3.78	40	6.02	3.72
16	5.41	4.50	41	5.40	4.44
17	5.07	4.00	42	5.78	3.90
18	6.35	3.70	43	5.05	3.82
19	6.11	3.96	44	5.85	3.51
20	6.15	3.90	45	5.05	4.40
21	5.21	4.26	46	5.14	4.15
22	5.45	4.02	47	5.36	4.10
23	6.44	4.04	48	6.05	3.96
24	5.14	4.06	49	5.21	4.02
25	5.59	4.20	50	6.01	4.41

**Table 5:** Statistical table of nursing satisfaction of the test group and the control group.

No.	Control group (%)	Test group (%)	No.	Control group (%)	Test group (%)
1	67.23	79.07	26	77.66	88.51
2	80.11	87.89	27	83.27	83.97
3	79.76	84.06	28	65.86	77.84
4	71.66	88.80	29	67.62	90.63
5	68.03	81.49	30	65.69	92.63
6	81.38	86.85	31	68.83	77.46
7	71.29	77.49	32	70.74	83.15
8	84.42	79.19	33	76.17	86.94
9	74.43	92.60	34	75.09	84.21
10	67.92	82.52	35	83.82	80.79
11	77.90	91.98	36	74.59	93.62
12	82.39	75.18	37	66.53	89.57
13	70.79	83.54	38	79.59	92.04
14	69.23	79.27	39	81.77	84.40
15	74.14	94.76	40	71.77	75.13
16	78.72	86.69	41	74.66	90.07
17	82.06	76.16	42	76.47	75.50
18	83.42	77.39	43	71.38	82.21
19	68.46	90.69	44	82.78	89.37
20	66.22	88.43	45	78.49	75.14
21	69.87	84.73	46	78.63	83.45
22	74.90	82.08	47	66.96	90.79
23	73.21	92.53	48	80.04	94.61
24	79.89	79.47	49	80.13	80.74
25	78.96	81.14	50	77.87	81.69

## Data Availability

The data used to support the findings of this study are included within the article.
